# Clinical Application of Spiral CT Reconstruction Imaging in Patients with Tracheal Stenosis before Anesthesia

This article has been retracted.

**DOI:** 10.1155/2022/9633527

**Published:** 2022-08-29

**Authors:** Shijie Dai, Yingying Yao, Daolin Xia

**Affiliations:** ^1^Department of Anesthesiology, The Fifth People's Hospital of Wuxi, Wuxi, Jiangsu, China; ^2^Department of Anesthesiology, Xuzhou Municipal Hospital Affiliated to Xuzhou Medical University, Xuzhou 221116, China; ^3^Department of Anesthesiology, Xuyi People's Hospital, Xuyi, Jiangsu 211700, China

## Abstract

In order to solve the problem of CT reconstruction imaging, this paper presents a study on the clinical application of preanesthesia in patients with tracheal stenosis. Patients with tracheal stenosis and multislice spiral CT virtual endoscopy (CTVE) were diagnosed, and their application effects were analyzed. *Methods*. 60 patients with tracheal stenosis were selected for clinical observation. The patients were given tracheal stenosis examination and multislice spiral CT virtual endoscopy. The examination results of the two groups were compared and analyzed by statistical methods. *Results*. There was no significant difference in the detection rate, sensitivity, accuracy, and specificity between the two groups (*P* > 0.05). *Conclusion*. Multislice spiral CT virtual endoscopy combined with a fiberoptic bronchoscope for clinical diagnosis of tracheal stenosis can complement each other. Combined use can effectively improve the detection consistency, and is safe and reliable. It can be used as an effective means for the diagnosis of tracheal stenosis.

## 1. Introduction

The causes of tracheal stenosis are complex, which are related to intratracheal tuberculosis, external compression of the trachea, and intratracheal benign and malignant tumors. In recent years, with the development of medical imaging technology, spiral CT reconstruction imaging has played an important role in the diagnosis of tracheal stenosis. It can intuitively and clearly understand the anatomical relationship between the airway and surrounding tissues, and provide an important reference for disease diagnosis and treatment. The study found that for patients with tracheal stenosis, the risk of general anesthesia with endotracheal intubation is high, and may affect the quality of anesthesia and surgical effect. Therefore, before operation, the airway condition should be evaluated to ensure the effect of operation and anesthesia. Spiral CT reconstruction imaging has a positive significance in assessing the degree of airway stenosis due to its high-density resolution and fast imaging speed, and the use of reconstruction technology can reduce the impact of overlapping projection and external tissue structure. Therefore, this article will apply spiral CT reconstruction imaging analysis in anesthesia of patients with tracheal stenosis, and analyze its application value, as shown in Figure 1.

## 2. Literature Review

Tracheal stenosis is a common clinical symptom in clinics. It is mainly caused by benign and malignant tumor in the trachea and bronchus, tuberculosis in the airway, external compression of the trachea, and so on. With the development of medical imaging, multislice spiral CT reconstruction technology can intuitively and clearly display the three-dimensional anatomical relationship of the human airway and adjacent tissues, and has obvious advantages in diagnosing the causes of tracheal stenosis or providing relevant valuable imaging data. Patients undergoing general anesthesia with endotracheal intubation, if complicated with tracheal stenosis, may affect the quality of anesthesia to a certain extent, thus reducing the surgical effect. It is necessary to evaluate the 'patients' airway before operation, so as to improve the quality of anesthesia and ensure the operation effect. Multislice spiral CT has a fast imaging speed and high-density resolution. Its various postprocessing techniques can be free from the influence of the tissue structure outside the slice, without overlapping projection, and can reconstruct the image in the later stage. The degree of airway stenosis of patients can be evaluated before surgery” [1].

## 3. Research Methods

### 3.1. General Information

Forty-seven patients who underwent general anesthesia with endotracheal intubation in a hospital from February 2017 to January 2018 were selected for retrospective analysis. Among the 47 patients, there were 29 male patients and 18 female patients, aged from 18 to 74 years, with an average age of 36.74 ± 6.15 years; weight 47∼74 kgs, an average weight of 58.45 ± 5.93 kgs; All the 47 patients underwent general anesthesia with endotracheal intubation. Before operation, the X-ray plain film showed that 21 cases had tracheal compression stenosis, and 26 cases had self-reported dyspnea and restriction.

### 3.2. Inclusion Criteria

(1) No other serious respiratory diseases; (2) all patients underwent multislice spiral CT examination; (3) clinical and imaging data are complete [2].

### 3.3. Exclusion Criteria

(1) Patients with severe heart and lung dysfunction; (2) contraindications of CT examination, such as spatial claustrophobia; (3) lactating women and pregnant women; (4) those who did not undergo tracheal intubation and general anesthesia; (5) those who did not cooperate with the study examiner [3].

### 3.4. Image Inspection

Before the examination, the patients need to remove the metal ornaments on their clothes or wear to avoid artifact interference affecting the imaging quality. At the same time, all patients should undergo the iodine allergy test. Only those who pass the test can undergo the multislice spiral CT examination. The equipment adopts spiral CT. First, perform CT plain scanning. The patient is in the supine position, and the arms are placed on both sides of the body. The scanning range is from the ear eyebrow line to the lower edge of the 7th cervical vertebra. The way of entering the bed is as follows: head first and foot second. The tube voltage is 120 kV, the tube current is 195 mA, the spacing is 5 mm, and the scanning layer thickness is 5 mm. After scanning, the scanned image is transferred to the computer background for reconstruction. The reconstruction layer is 1.25 mm thick. Multiplane reconstruction technology, simulated airway mirror technology, and volume reconstruction technology were used [4–6].

### 3.5. Image Processing

According to CT images, the degree of tracheal stenosis was classified as follows: grade I: the degree of airway obstruction was less than 70%; grade II: airway obstruction 70% ∼ 90%; grade III: the degree of airway obstruction is greater than 90%; grade IV: complete airway obstruction. The CT workstation was equipped with an electronic device to measure the following: (1) the cross-sectional area and diameter of the narrower position of the compressed trachea; (2) the distance between the end of compressed tracheal stenosis and the cricoid cartilage; (3) the length of trachea compression stenosis; (4) the cross-sectional area and diameter of the compressed gas tube at the end [7].

### 3.6. Statistical Treatment

All the data in this study were tested by SPSS18.0 statistical software. The measurement data were statistically described by $\bar{\chi }$ ± *s*. The average age of patients and other counting data were described by the adoption rate and constituent ratio. The difference was statistically significant with *P* < 0.05 [8].

### 3.7. Measurement of Cross-Sectional Area and Diameter of the Most Severe Tracheal Stenosis by Spiral CT Reconstruction

The minimum cross-sectional area of the most severe tracheal stenosis was 0.69 cm, the maximum was 1.46 cm, and the average cross-sectional area was 2.06 ± 1.54 cm; the minimum cross-sectional diameter of the most severe tracheal stenosis was 4.42 mm, the maximum was 9.53 mm, and the average cross-sectional area was 6.43 ± 1.27 mm, as shown in Table 1.

### 3.8. Evaluation of Tracheal Stenosis by Spiral CT Reconstruction

After sorting out the imaging data of 48 patients, it was found that 28 patients with grade I tracheal stenosis and 19 patients with grade II tracheal stenosis were assessed by spiral CT reconstruction imaging. The diameter of the trachea in the noncompressed position was 10.14∼16.75 mm, with an average diameter of 13.01 ± 2.12 mm; the minimum length of stenosis was 2.71 cm and the maximum was 6.09 cm, with an average of 4.12 ± 0.69 cm; the cross-sectional area of the trachea at the unpressurized position was 1.20∼2.95 cm, with an average of 1.98 ± 0.31 cm; the minimum distance between the end of tracheal stenosis and cricoid cartilage was 4.81 cm, the maximum was 7.32 cm, and the average value was 5.79 ± 0.62 cm. According to the image evaluation of 47 cases of spiral CT reconstruction, there was no intubation failure during general anesthesia with endotracheal intubation. The success rate was 100%. During anesthesia, the oxygen saturation detection was 95∼100%, and end expiratory carbon dioxide detection was 3.50∼5.51 kPa, as shown in Table 2.

Esophageal cancer, thyroid cancer, abscess, hematoma, tracheal tumor, and tracheomalacia can all cause bronchial stenosis. The clinical manifestations of patients with airway stenosis are shortness of breath and dyspnea, as well as cough, expectoration, and other clinical symptoms. Clinical auscultation can find that the patient's respiratory sound is low or disappeared, and there are dry and wet rales at the same time. At present, the clinical examination of airway stenosis mainly depends on auxiliary examination, including clinical physical examination and imaging examination. The physical examination method is as follows: when the patient is silent, his mouth and tongue is opened to the maximum, and Mallampati airway classification is carried out according to the pharyngeal structure seen, but many scholars believe that the examination method is too subjective to assess the degree of stenosis, which is directly related to the doctor's experience and cannot be accurate. The patient's gas-to-stenosis situation is comprehensively observed [9–11]. Some scholars have discussed the value of the three-dimensional reconstruction of multislice spiral CT in the diagnosis of suspected etiology of asthma in children. They believe that some patients with airway diseases have no specificity in clinical symptoms and signs, and imaging examination images, which increases the difficulty of diagnosis. However, MSCT three-dimensional airway reconstruction technology can clearly display the structure of the airway and its surrounding tissues, which has extremely important clinical value in identifying the etiological diagnosis of children's wheezing or asthmatic diseases and reducing misdiagnosis [12]. Other scholars collected the clinical data of 15 patients with tracheal stenosis. All patients were diagnosed by spiral CT reconstruction imaging and observed the relevant diagnosis. The results showed that the application of spiral CT reconstruction imaging in anesthesia of patients with tracheal stenosis could help clinical treatment [13]. This group studied and analyzed the clinical application value of spiral CT reconstruction before anesthesia in patients with tracheal stenosis. The results showed that spiral CT reconstruction before anesthesia can effectively measure and evaluate tracheal stenosis. The minimum cross-sectional area of the most severe tracheal stenosis was 0.79 cm and the maximum was 1.36 cm. The average cross-sectional area of the most severe tracheal stenosis was 6.53 ± 1.17 mm. In the grading of tracheal stenosis assessed by spiral CT reconstruction imaging, 28 cases had grade I tracheal stenosis and 19 cases had grade II tracheal stenosis. The diameter of the trachea at the noncompressed position, the length of the stenosis segment, the cross-sectional area of the trachea at the noncompressed position, and the minimum distance between the end of the stenosis segment of the trachea and the cricoid cartilage could be directly measured to obtain data. Spiral CT reconstruction imaging technology is one of the most widely used examination methods in clinics at present. It can measure the number, location, morphological characteristics, and the thickness of the bronchial wall more intuitively, quantitatively, and in multiple parts. Compared with bronchoscopy, it is noninvasive and convenient, especially for elderly and infant patients. In the observation of the anesthesia effect, according to the evaluation of 47 cases of spiral CT reconstruction image, there was no intubation failure during general anesthesia of endotracheal intubation, and the success rate was 100%. The detection of oxygen saturation and end expiratory carbon dioxide during anesthesia were within the normal range, indicating that the spiral CT reconstruction image before anesthesia can effectively measure and evaluate tracheal stenosis [14–16]. Spiral CT has a good representation of the complete anatomical surface of the trachea through reconstruction. It can directly measure the internal diameter of organs. At the same time, combined with the relevant data of the narrowest part of the airway, it can measure the degree and diameter of the patient's trachea stenosis, simulate the original image, fully display the structure of the inner surface of the trachea and the lumen structure, and obtain more reliable information [17].

## 4. Experiment and Research

The method of spiral CT reconstruction imaging refers to the use of computer postprocessing technology to do three-dimensional reconstruction of the airway on the basis of thin-layer volume data acquisition of spiral CT. Various two-dimensional (2D) and three-dimensional (3D) tracheobronchial images can be reconstructed to truly display the lesions. CT reconstruction of trachea and bronchus can provide an accurate basis for the display and diagnosis of bronchial foreign bodies, new organisms, tracheal stenosis, and other diseases [18].

60 patients with clinically diagnosed tracheal stenosis admitted to a hospital from October 2009 to July 2012 were selected for a retrospective analysis. The inclusion criteria were as follows: previous history of tuberculosis or sputum examination within the last 3 months. The examination results showed that the patients' acid-fast bacilli were positive. Among them, there were 24 male patients and 36 female patients. The youngest was 15 years of age and the oldest was 70 years of age. The average age was 45.8 + 4.6 years old. The main clinical manifestations were cough, hemoptysis, expectoration, night sweats, and chest pain; in addition, all patients were given X-ray examination. The X-ray results of 53 patients showed pulmonary lesions, 17 patients showed obstructive emphysema, 12 patients showed atelectasis, and 7 patients showed obstructive pneumonia [19, 20], as shown in Table 3.

### 4.1. Multislice Spiral CT Virtual Endoscopy Processing Method

Select the 16-layer spiral CT machine, make the patient take the supine position, and then raise both hands to scan the patient's lungs, starting from the double lung tips and to the bottom of the patient's lungs. During scanning, the scanning parameters of the spiral CT machine are as follows: tube voltage and tube current are respectively l20 kV and 200 mAs. The scanning method is continuous volume high-resolution scanning, with a layer thickness of 0.6 mm. On the postprocessing workstation, multislice spiral CT virtual endoscopy postprocessing is performed on the image, and the scanning results are recorded in detail [21].

### 4.2. Examination Method for Tracheal Stenosis

Within 3 days before and after giving the patients CT examination, the patients were examined for tracheal stenosis. At the same time, the endobronchial tissues of the patients were selected, and the endobronchial tissues were biopsied. Then, sputum smears and pictures of bronchial lavage fluid or fiberoptic bronchoscope brush films were made. The acid-fast bacilli level in the films was examined, and the examination data were recorded as the gold standard [22].

### 4.3. Image Evaluation

The blind method was used to make independent diagnosis on CT images. Only when the diagnostic results are consistent can they be regarded as CT diagnostic results.

### 4.4. Statistical Methods

SPSS15.0 software was used for statistical analysis of the experimental data. The *T*-test was used. The Chi square test was used to compare the counting data. The difference was statistically significant with *P* < 0.05 [23].

### 4.5. Results

#### 4.5.1. Analysis of the Diagnostic Results of the Two Groups

In multi-slice spiral CT virtual endoscopy, 52 patients were diagnosed as tracheal stenosis, 3 patients were diagnosed as central lung cancer, 2 patients were diagnosed as inflammatory lesions, and the other 3 patients could not be judged. Among the 52 patients with tracheal stenosis diagnosed by multislice spiral CT virtual endoscopy, the CT images mainly showed homogeneous stenosis, occlusion, and heterogeneous stenosis, with a total of 106 lesions. Among them, 24 were homogeneous stenosis, 12 were bronchial occlusion, and 70 were heterogeneous stenosis; in the fiberoptic bronchoscopy, 1 was homogeneous stenosis, 1 was bronchial occlusion, and 2 were heterogeneous stenosis, accounting for 5.7%. The multislice spiral CT virtual endoscopy image showed bronchial changes in the distant lung segment of bronchial stenosis [24].

In the examination of tracheal stenosis, 54 patients had tracheal stenosis, 3 patients had inflammatory lesions, and 3 patients had central lung cancer, as shown in Table 4.

There was no significant difference between the two groups (*P* > 0.05). The accuracy, sensitivity, and specificity of multislice spiral CT virtual endoscopy were 90.0%, 92.3%, and 66.7%, respectively.

#### 4.5.2. Analysis of the Results of the Two Groups

The main subtypes of tracheal stenosis were hyperemia edema type, ulcer granulation type, infiltration proliferation type, and scar stenosis type, with 37, 25, 24, and 23 sites, respectively, and a total of 109 sites. Among them, in the multislice spiral CT virtual endoscopy, a total of 102 cases were consistent with tracheal stenosis, and the main noncompliance was the hyperemia edema type and infiltration proliferation type, with 5 cases and 2 cases, respectively, accounting for 6.4%. The main manifestations of multislice spiral CT virtual endoscopy typing are shown in Table 5.

### 4.6. Complications Seen by Multislice Spiral CT Virtual Endoscopy

In multislice spiral CT virtual endoscopy, there were 12 patients with obstructive atelectasis, 9 patients with obstructive pneumonia, and 7 patients with obstructive emphysema.

### 4.7. Discussion

Clinically, tracheal stenosis is usually classified into the following four types: hyperemia and edema, ulcer granulation, infiltration and proliferation, and scar stenosis. The disease progresses slowly but has many clinical symptoms that lack specificity. Therefore, it is difficult to make a definite diagnosis in clinical diagnosis. The missed diagnosis and misdiagnosis of tracheal stenosis may lead to bronchofibrostenosis, and then lead to atelectasis and secondary lung infection. Accurate diagnosis of tracheal stenosis plays a vital role in the clinical treatment and curative effect of tracheal stenosis [25].

Multi-slice spiral CT virtual endoscopy is a new method combining computer simulation and CT volume scanning. The imaging basis of this method is mainly to reconstruct the scanned data into a three-dimensional image through continuous volume scanning of multislice spiral CT. On this basis, the transparency and the threshold of the CT value are adjusted, and then, the object screen distance, video screen distance, light, and perspective direction are properly adjusted by using the calculation connection technology. At the same time, the artificial pseudo-color is added, and finally the scanning effect similar to that of a fiber endoscope can be obtained.

It can be seen from Table 5 of the results that in multislice spiral CT virtual endoscopy, the manifestations of bronchial tuberculosis are mainly uneven stenosis, mainly because the resolution of this examination method is lower than that of fiberoptic bronchoscopy. Some cases show cauliflower-like new organisms, and nipple and granulation hyperplasia under a fiberoptic bronchoscope, but also uneven stenosis in multislice spiral CT virtual endoscopy. In this study, 23 of the multislice spiral CT virtual endoscopy were homogeneous stenosis, while the fiberoptic bronchoscope was mainly infiltrative proliferative and hyperemic edema. The detection rates of these two types were more consistent. In the multislice spiral CT virtual endoscopy, the proportion of complete obstruction was 10.8%. Under the fiberoptic bronchoscope, there were 2 eccentric stenoses, mainly because when the human bronchus reached a certain degree of stenosis, there would be a volume defect, which was mainly manifested as interruption. At this time, when the multi-slice spiral CT virtual endoscopy was used, the image would show complete occlusion.

## 5. Conclusion

Spiral CT airway reconstruction imaging can display the shape and changes of the airway in multiple planes and different angles. With the advantage of high resolution, the image quality in the display of airway stenosis is high. In conclusion, spiral CT reconstruction imaging before anesthesia can effectively measure and evaluate tracheal stenosis, provide relevant data for clinical general anesthesia with endotracheal intubation, and ensure the success rate of anesthesia at one time. Multi slice spiral CT virtual endoscopy has no obvious contraindications, will not cause trauma to patients, and will not have adverse sequelae. In addition, this diagnostic method can further observe the long axis range and stenosis degree of the stenotic segment in the patient's focus, effectively understand the lung tissue around the patient's focus and the occurrence of complications, effectively determine the lesion range, and observe the extraluminal conditions, which are better than the examination of tracheal stenosis. Therefore, in the clinical diagnosis of tracheal stenosis, multislice spiral CT virtual endoscopy combined with tracheal stenosis can play a certain role in the diagnosis.

## Figures and Tables

**Figure 1:** Spiral CT reconstruction in tracheal stenosis.

**Table 1:** Cross-sectional area and diameter of the most severe tracheal stenosis measured by spiral CT reconstruction imaging.

Category	Range	Average value
Cross load area	0.78–1.26	1.25–0.55
Diameter	3.52–8.36	6.85–1.27

**Table 2:** Analysis of trachea stenosis at the heaviest compression part and end compression part of the trachea.

Project	Number of columns	The most serious part	End compression part
Cross load area	48	1.06–0.56	1.89–0.42
Diameter	18	6.25–2.10	13.25–2.88

**Table 3:** Comparison of 16 slice spiral CTVB and FB in the lesion group.

	Block	Stiff and narrow	Cauliflower-like new organism
Closed race	5	7	5
Narrow	2	0	2
Seize a seat	0	0	3

**Table 4:** Analysis of diagnosis results of the two groups.

CTVE diagnostics	Endobronchial tuberculosis	Nonendobronchial tuberculosis	Total
Endobronchial tuberculosis	60		63
Nonendobronchial tuberculosis	5	5	10
Total	55	7	62

**Table 5:** Classification performance of multislice spiral CT under virtual endoscopy.

Project	Hyperemic edematous type	Infiltrative proliferative type	Epileptic scar stenosis	Total
Complete closure	2	5	4	11
Uniform stenosis	11	3	6	20
Nonuniform stenosis	31	5	10	46
Total	44	13	20	77

## Data Availability

The data used to support the findings of this study are available from the corresponding author upon request.
